RETRACTED

# Clinical features of 375 COVID-19 cases imported from Russia through the Suifenhe port and countermeasures

**DOI:** 10.1371/journal.pone.0261437

**Published:** 2021-12-16

**Authors:** Kai Kang, Yi Yang, Xiangdong Guan, Yan Kang, Mingyan Zhao, Jianbo Yu, Xiqiu Zeng, Fengjie Xie, Guolin Chen, Kaijiang Yu

**Affiliations:** 1 Department of Critical Care Medicine, The First Affiliated Hospital of Harbin Medical University, Harbin, Heilongjiang Province, China; 2 Department of Critical Care Medicine, Zhongda Hospital, School of Medicine, Southeast University, Nanjing, Jiangsu Province, China; 3 Department of Critical Care Medicine, The First Affiliated Hospital of Sun Yat‑sen University, Guangzhou, Guangdong Province, China; 4 Department of Critical Care Medicine, West China Hospital, Sichuan University, Chengdu, Sichuan Province, China; 5 Department of Critical Care Medicine, The Hongqi Hospital Affiliated Mudanjiang Medical University, Mudanjiang, Heilongjiang Province, China; 6 The Kangan Hospital, Mudanjiang, Heilongjiang Province, China; 7 Department of Infectious Disease, The First Affiliated Hospital of Harbin Medical University, Harbin, Heilongjiang Province, China; 8 Institute of Critical Care Medicine in Sino Russian Medical Research Center of Harbin Medical University, Harbin, China; Konkuk University, REPUBLIC OF KOREA

## Abstract

**Background and objectives:**

At present, the focus of the fighting against COVID-19 in China is shifting to strictly prevent the entrance of cases from abroad and disease transmission. Therefore, it is extremely urgent to better understand the clinical features of imported cases from overseas countries, which is conductive to formulate the corresponding countermeasures. This study aimed to describe the clinical features of COVID-19 cases imported from Russia through the Suifenhe port, in order to identify baseline and clinical data associated with disease progression and present corresponding countermeasures.

**Methods:**

All COVID-19 cases imported from Russia through the Suifenhe port were included in this retrospective study. According to the “Diagnosis and Treatment Protocol for Novel Coronavirus Pneumonia (seventh edition)”, imported COVID-19 cases were divided into asymptomatic infection, mild, moderate, severe, and critical groups. Baseline and clinical data, including age, gender, comorbidities, disease severity, symptoms at onset, body temperature, white blood cell (WBC) count, lymphocyte (LYMPH) count, lymphocyte percentage (LYM%), C-reactive protein (CRP), oxygenation index (OI), and the use therapeutic modalities were obtained on admission, and then compared between groups.

**Results:**

A total of 375 COVID-19 cases imported from Russia through Suifenhe port were included, of whom the asymptomatic infection, mild, moderate, severe, and critical groups accounted for 4.0%, 13.9%, 75.5%, 5.3%, and 1.3%, respectively. The majority of the imported COVID-19 cases were men (61.9%) with a median age of 38.72 years who had no comorbidity (87.7%). Nearly one-third of them (33.1%) were asymptomatic at onset, and common initial symptoms included fever (36.5%), cough (36.0%), pharyngeal discomfort (12.3%), expectoration (8.0%), and chest tightness (5.3%). In total, 180 (48%) and 4 (1.1%) enrolled imported cases received nasal tube oxygen inhalation therapy and high-flow oxygen absorption, respectively; the remaining patients did not undergo oxygen therapy. The values of age, body temperature, WBC, LYMPH, LYM%, CRP, and OI were 38.72 ± 10.50, 35.10 ± 7.92, 5.59 ± 1.97, 1.67 ± 0.68, 31.05 ± 10.22, 8.00 ± 14.75, and 389.03 ± 74.07, respectively. Gender, age, LYMPH, LYM%, symptoms at onset, cough, fever, other rare symptoms, and oxygen therapy showed significant differences between groups (P = 0.036, < 0.001, < 0.001, < 0.001, < 0.001, < 0.001, < 0.001, = 0.045, < 0.001, respectively).

RETRACTED

**Conclusions:**

Compared with domestic confirmed patients, COVID-19 patients who arrived at China from Russia through the Suifenhe port had significantly different clinical features, and the differences in gender, age, LYMPH, LYM%, symptoms at onset, cough, fever, other rare symptoms, and oxygen therapy between groups were statistically significant. Therefore, detailed and comprehensive countermeasures were developed to manage and prevent another outbreak based on these clinical features.

## Introduction

Coronavirus disease 2019 (COVID-19) is wreaking havoc around the world, with the mutations of severe acute respiratory syndrome coronavirus type 2 (SARS-CoV-2) aggravating the current situation even more [1, 2]. Coronavirus disease 2019 (COVID-19) outbreak has been far more devastating than expected, showing no signs of slowing down at present. COVID-19 has led to more deaths than the sum of severe acute respiratory syndrome CoV (SARS-CoV) and Middle East respiratory syndrome CoV (MERS-CoV). The case-fatality rate of COVID-19 as reported previously varied from 3.77% to 28% in Wuhan (epicenter area) [3–10], and this percentage was significantly higher than that in other non-epicenter areas of China [9, 11]. COVID-19 is spreading and wreaking havoc worldwide, especially in the United States and Europe [12], imposing huge challenges to healthcare systems and economic development. As the number of domestic confirmed cases continue to decline, the prevention and control of COVID-19 are on the verge of victory in China. For the next step, the focus of epidemic prevention and management has been shifted to the strict prevention of imported cases from abroad, however, little is known about the clinical features of imported COVID-19 cases from overseas countries. With the surge of returnees from overseas, this task has become extremely arduous, especially at the Suifenhe port, the only remaining Sino-Russian land port in Heilongjiang province (China), which has a long history and resident population of only 70,000. Several national and provincial experts and medical teams have rushed to Suifenhe and Mudanjiang to relieve medical stress.

RETRACTED

With the increasing number of cases imported from Russia through the Suifenhe port, it is highly essential to understand the clinical features of such cases, identify baseline and clinical data associated with disease progression, and formulate corresponding countermeasures to prevent the spread of COVID-19. The comparison of imported cases with differences in disease severity can result in identification of baseline and clinical data associated with disease progression to facilitate the early diagnosis and intervention of risky imported patients, and thereby reduce the incidence of severe or critical cases. Previous research showed that the mortality rate of critically ill COVID-19 patients even reached 60% [13]. Although the recent increase of imported cases from Russia slowed down due to the temporary closure of the Suifenhe port, an improper response may result in disastrous consequences.

This study aimed to describe clinical features of COVID-19 cases imported from Russia through the Suifenhe port, identify baseline and clinical data associated with disease progression, and present corresponding countermeasures based on findings of this study.

## Methods

### Study design

This retrospective study included all imported COVID-19 cases from Russia through the Suifenhe port who were treated in Suifenhe square cabin hospital, Mudanjiang Ankang hospital, and Hongqi Hospital Affiliated Mudanjiang Medical University due to differences in disease severity. According to the “Diagnosis and Treatment Protocol for Novel Coronavirus Pneumonia (seventh edition)”, imported COVID-19 cases were divided into asymptomatic infection, mild, moderate, severe, and critical groups. Baseline and clinical data were collected on admission and then compared between groups. This study was approved by the Ethics Committee of the First Affiliated Hospital of Harbin Medical University (Harbin, China). The informed consent was waived by the ethics committee for the observational and retrospective nature.

### Study population

In this retrospective study, the inclusion criterion was confirmed as imported COVID-19 cases from Russia through the Suifenhe port. All enrolled imported COVID-19 patients were addressed using similar treatment regimens according to the “Diagnosis and Treatment Protocol for Novel Coronavirus Pneumonia (seventh edition)”.

RETRACTED

### Diagnosis of COVID-19

All enrolled imported cases were diagnosed as severe acute respiratory syndrome coronavirus 2 (SARS-CoV-2) infection via nasopharyngeal swab nucleic acid amplification testing.

### Data acquisition

Baseline and clinical data, including age, gender, comorbidity, disease severity, symptoms at onset, body temperature, WBC, LYMPH, LYM%, CRP, OI on admission and therapeutic modalities, were collected from medical records. The members of our research team were blinded to patients’ personal data beyond the baseline and clinical data required for this study.

### Statistical analysis

SPSS 23.0 software (IBM, Armonk, NY, USA) was used to perform statistical analyses. The quantitative data were described as the mean ± standard deviation (SD), while the qualitative data were expressed as number. If the qualitative data met the predefined requirement, *χ*^*2*^ test was utilized; otherwise, the Fisher’s exact test was employed. Bonferroni correction test was used for making inter-group comparison. One-way analysis of variance (ANOVA) was employed for the comparison of normally distributed data between two groups, while the Kruskal-Wallis rank-sum test was utilized for comparing abnormally distributed data. Inter-group comparisons were made by using the least significant difference (LSD) method. P-value < 0.05 was considered statistically significant.

## Results

### Patients’ demographic and clinical characteristics

As shown in Table 1, a total of 375 imported COVID-19 cases from Russia through the Suifenhe port were included, of whom asymptomatic infection, mild, moderate, severe, and critical groups accounted for 4.0%, 13.9%, 75.5%, 5.3%, and 1.3%, respectively. The majority of the imported COVID-19 patients were men (61.9%), with a median age of 38.72 years old without comorbidity (87.7%). Imported cases with 1, 2, 3, and 4 types of comorbidities accounted for 10.1%, 1.1%, 0.8%, and 0.3% of the patients, respectively. Common comorbidities included hypertension (5.9%), diabetes (2.7%), coronary artery disease (1.6%), and hepatitis B virus (1.1%). Nearly one-third of imported patients (33.1%) were asymptomatic at onset, and common initial symptoms included fever (36.5%), cough (36.0%), pharyngeal discomfort (12.3%), expectoration (8.0%), and chest tightness (5.3%). In total, 180 (48%) and 4 (1.1%) enrolled imported patients received nasal tube oxygen inhalation therapy and high-flow oxygen absorption, respectively; the remaining patients did not obtain oxygen therapy. The values of age, body temperature, WBC, LYMPH, LYM%, CRP, and OI were 38.72 ± 10.50, 35.10 ± 7.92, 5.59 ± 1.97, 1.67 ± 0.68, 31.05 ± 10.22, 8.00 ± 14.75, and 389.03 ± 74.07, respectively (Table 2).

RETRACTED

**Table 1:** Patients’ demographic and clinical characteristics.

Characteristic	Classification	Frequency	Percentage
Disease severity	Asymptomatic infection	15	4.0
	Mild	52	13.9
	Moderate	283	75.5
	Severe	20	5.3
	Critical	5	1.3
Gender	Female	143	38.1
	Male	232	61.9
Number of comorbidities	0.00	329	87.7
	1.00	38	10.1
	2.00	4	1.1
	3.00	3	.8
	4.00	1	.3
Symptoms at onset	No	124	33.1
	Yes	251	66.9
Cough	No	240	64.0
	Yes	135	36.0
Fever	No	238	63.5
	Yes	137	36.5
Expectoration	No	345	92.0
	Yes	30	8.0
Pharyngeal discomfort	No	329	87.7
	Yes	46	12.3
Chest tightness	No	355	94.7
	Yes	20	5.3
Other rare symptoms	No	297	79.2
	Yes	78	20.8
Oxygen therapy	None	186	49.6
	Nasal tube oxygen inhalation therapy	180	48.0
	High-flow oxygen absorption	4	1.1

**Table 2:** Demographic and clinical data of imported COVID-19 cases from Russia through the Suifenhe port.

	N	Min	Max	Mean	SD	P25	P50	P75
Age	375	14.00	66.00	38.72	10.50	31.00	39.00	47.00
Body temperature	375	35.50	39.50	35.10	7.92	36.30	36.60	37.10
WBC	375	2.17	14.30	5.59	1.97	4.12	5.15	6.75
LYMPH	375	0.36	4.55	1.67	0.68	1.23	1.58	2.05
LYM%	375	3.63	64.90	31.05	10.22	23.90	30.90	38.30
CRP	372	1.70	105.04	8.00	14.75	1.70	1.70	7.80
OI	276	50.00	666.00	389.03	74.07	362.25	398.00	428.00

### Comparison of imported COVID-19 cases with different levels of disease severity

As summarized in Table 3, an inter-group comparison showed that the proportion of male patients in the asymptomatic infection group was higher than that in the mild group (P = 0.036). As shown in Tables 3 and 4, the differences in age between groups were statistically significant (P < 0.001), except for the asymptomatic infection and mild groups, indicating that age increased as the disease progressed. The differences in LYMPH between groups were statistically significant (P < 0.001), except for the mild and moderate groups, manifesting that LYMPH decreased as the disease progressed. LYM% in the critical and severe groups was significantly lower than that in the asymptomatic infection, mild, and moderate groups (P < 0.001). As presented in Table 5, cough, fever, and oxygen therapy showed significant differences between groups (P < 0.001, < 0.001, < 0.001, respectively). The differences in symptoms at onset between groups were statistically significant (P < 0.001), except for the moderate group and the critical or severe group, reflecting the enhancement of symptoms at onset as the disease progressed. The incidence of other rare symptoms in critical or severe group was significantly higher than that in mild group (P = 0.045).

RETRACTED

**Table 3:** Comparison of gender, comorbidities, age, LYMPH, and LYM% between groups with different levels of disease severity.

		Asymptomatic infection (N = 15)	Mild (N = 52)	Moderate (N = 283)	Critical or Severe (N = 25)	*X2*	*P*
Gender	Female	1	25	108	9	8.523	0.036
	Male	14	27	175	16		
Comorbidities	No	14	45	251	19	3.366	0.282
	Yes	1	7	32	6		
Age (years old)		30.67 ± 8.85	34.81 ± 9.20	39.27 ± 10.42^a^^b^	45.56 ± 9.55^a^^b^^c^	9.782	<0.001
LYMPH		2.49 ± 0.49	1.84 ± 0.68^a^	1.66 ± 0.63^a^	0.88 ± 0.44^a^^b^^c^	23.661	<0.001
LYM (%)		35.85 ± 5.72	32.81 ± 9.23	31.80 ± 9.69	15.96 ± 7.61^a^^b^^c^	24.082	<0.001

^a, b^ and ^c^ represent significant differences compared with the asymptomatic infection, mild, and moderate groups, respectively.

**Table 4:** Inter-group comparisons of age, LYMPH, and LYM% between groups with different levels of disease severity.

Dependent variable	(I) Group	(J) Group	Mean difference (I-J)	Standard error	Significance	95% confidence interval	
						Lower limit	Upper limit
Age (years old)	Asymptomatic infection	Mild	-4.14103	2.97445	.165	-9.9899	1.7079
		Moderate	-8.59835*	2.68897	.002	-13.8859	-3.3108
		Critical or Severe	-14.89333*	3.31460	.000	-21.4111	-8.3756
	Mild	Asymptomatic infection	4.14103	2.97445	.165	-1.7079	9.9899
		Moderate	-4.45733*	1.53124	.004	-7.4683	-1.4463
		Critical or Severe	-10.75231*	2.46996	.000	-15.6092	-5.8954
	Moderate	Asymptomatic infection	8.59835*	2.68897	.002	3.3108	13.8859
		Mild	4.45733*	1.53124	.004	1.4463	7.4683
		Critical or Severe	-6.29498*	2.11753	.003	-10.4588	-2.1311
	Critical or Severe	Asymptomatic infection	14.89333*	3.31460	.000	8.3756	21.4111
		Mild	10.75231*	2.46996	.000	5.8954	15.6092
		Moderate	6.29498*	2.11753	.003	2.1311	10.4588
LYMPH	Asymptomatic infection	Mild	.65218*	.18231	.000	.2937	1.0107
		Moderate	.83093*	.16482	.000	.5068	1.1550
		Critical or Severe	1.61733*	.20316	.000	1.2178	2.0168
	Mild	Asymptomatic infection	-.65218*	.18231	.000	-1.0107	-.2937
		Moderate	.17875	.09386	.058	-.0058	.3633
		Critical or Severe	.96515*	.15139	.000	.6675	1.2628
	Moderate	Asymptomatic infection	-.83093*	.16482	.000	-1.1550	-.5068
		Mild	-.17875	.09386	.058	-.3633	.0058
		Critical or Severe	.78640*	.12979	.000	.5312	1.0416
	Critical or Severe	Asymptomatic infection	-1.61733*	.20316	.000	-2.0168	-1.2178
		Mild	-.96515*	.15139	.000	-1.2628	-.6675
		Moderate	-.78640*	.12979	.000	-1.0416	-.5312
LYM (%)	Asymptomatic infection	Mild	3.03705	2.75009	.270	-2.3707	8.4448
		Moderate	4.04349	2.48614	.105	-.8452	8.9322
		Critical or Severe	19.88867*	3.06458	.000	13.8625	25.9148
	Mild	Asymptomatic infection	-3.03705	2.75009	.270	-8.4448	2.3707
		Moderate	1.00644	1.41574	.478	-1.7774	3.7903
		Critical or Severe	16.85162*	2.28365	.000	12.3611	21.3421
	Moderate	Asymptomatic infection	-4.04349	2.48614	.105	-8.9322	.8452
		Mild	-1.00644	1.41574	.478	-3.7903	1.7774
		Critical or Severe	15.84518*	1.95780	.000	11.9954	19.6950
	Critical or Severe	Asymptomatic infection	-19.88867*	3.06458	.000	-25.9148	-13.8625
		Mild	-16.85162*	2.28365	.000	-21.3421	-12.3611
		Moderate	-15.84518*	1.95780	.000	-19.6950	-11.9954

* Indicates significance at the 5% level

RETRACTED

**Table 5:** Comparison of symptoms at onset and oxygen therapy between groups with different levels of disease severity.

		Mild	Moderate	Critical or Severe	*Χ* ^*2*^	*P*
Symptoms at onset	No	31	76	2	28.469	<0.001
	Yes	21	207	23		
Cough	No	44	173	8	21.000	<0.001
	Yes	8	110	17		
Fever	No	47	169	7	30.657	<0.001
	Yes	5	114	18		
Expectoration	No	50	260	20	5.122	0.059
	Yes	2	23	5		
Pharyngeal discomfort	No	42	249	23	2.416	0.289
	Yes	10	34	2		
Chest tightness	No	50	268	22	2.317	0.308
	Yes	2	15	3		
Other rare symptoms	No	44	223	15	6.169	0.045
	Yes	8	60	10		
Oxygen therapy	No	45	126	0	54.798	<0.001
	Yes	7	152	25		

## Discussion

COVID-19 has been confirmed to be caused by SARS-CoV-2 infection [14] and has complex clinical manifestations ranging from asymptomatic infection to fatal critical illnesses that mostly present as acute respiratory distress syndrome (ARDS) and require mechanical ventilation support [15, 16]. An excessive and uncontrolled response to SARS-CoV-2 infection can induce injury or failure of different vital organs in the clinic. At present, COVID-19 is mainly diagnosed by real-time polymerase chain reaction (RT-PCR) detection of SARS-CoV-2 nucleic acids on oropharyngeal and/or nasopharyngeal swabs [17, 18], although there is a certain probability of false-positive and false-negative results [19–21]. If two consecutive negative results on a respiratory nucleic acid test (at an interval of at least 24 h) are used as the exclusion criterion, this may lead to missed diagnoses in approximately 10% of COVID-19 patients and the spread of the epidemic [22]. SARS-CoV-2 is characterised by its high infectivity, mainly through efficient human-to-human transmission [3, 8, 23, 24], especially among close contacts in closed environments. Since the Suifenhe port is the only remaining Sino-Russian land port in Heilongjiang province, it takes a long-time for returnees to return home by different modes of transportation, providing opportunities for infection with SARS-CoV-2.

To date, few studies have concentrated on foreign imported COVID-19 cases in China [24]. On April 2, 2020, four COVID-19 cases imported from Russia through the Suifenhe port were first confirmed. Since then, the number of patients has soared. For all patients with imported COVID-19 in the current study, their main occupations were as businessmen, students, migrant workers, and freelancers. Inevitably, different host characteristics will lead to different clinical features in the clinic. Huang et al. reported that 20 (49%) of the SARS-CoV-2-infected patients were aged 25–49 years, and 14 (34%) were aged 50–64 years, but Chen et al. reported that the mean age of the 99 patients was 55·5 years. The median age of the COVID-19 patients was 49·0 years (IQR 41·0–58·0) [3, 4]. However, from our study we can see that imported COVID-19 cases from Russia through the Suifenhe port were younger, with a median age of 38.72 years old, and had similar gender proportion and fewer comorbidities. The majority of the imported COVID-19 patients were men (61.9%) and had no comorbidities (87.7%). Rare comorbidities included chronic bronchitis (0.5%), chronic pharyngitis (0.5%), arrhythmia (0.5%), superficial gastritis (0.3%), nephritis (0.3%), chronic enteritis (0.3%), anxiety disorder (0.3%), acute lymphoblastic leukaemia (0.3%), thyroid carcinoma (0.3%), hypothyroidism (0.3%), cerebral infarction (0.3%), psoriasis (0.3%), and chronic urticaria (0.3%). The high proportion of asymptomatic carriers at onset (33.1%) in the present study indicated a remarkable difficulty in identification of SARS-CoV-2 infection patients only based on body temperature and chief complaints without further tests [2]. Available evidence showed that asymptomatic carriers, as a concern for prevention and control of COVID-19, were infectious to an extent.

RETRACTED

Symptoms observed at onset were variable. In addition to common symptoms, other rare initial symptoms included diarrhoea (4.53%), nasal congestion (2.93%), shortness of breath (2.40%), fatigue (2.13%), muscle soreness (1.33%), runny nose (1.33%), headache (1.33%), smell and/or taste disorder (1.33%), palpitation (0.80%), nausea (0.80%), panting (0.80%), shiver (0.53%), dizziness (0.53%), sneezing (0.53%), anorexia (0.27%), throat sore (0.27%), pectoralgia (0.27%), vomiting (0.27%), somnolence (0.27%), dyspnoea (0.27%), and general discomfort (0.27%). The incidence of symptoms at onset, fever, cough, and other rare symptoms significantly increased with disease progression. SARS-CoV-2 triggered a high prevalence of pneumonia rather than upper respiratory symptoms in infected patients, which was consistent with the results of the current study, due to the dense distribution of angiotensin-converting enzyme 2 (ACE2), a cellular receptor, in the lower respiratory tract. It is noteworthy that smell and/or taste disorders (STDs) are extremely frequent among overseas COVID-19 patients [25–27], even as a marker for SARS-CoV-2 infection [28], while those are rare in domestic patients. However, the underlying mechanism has still remained elusive. Due to high expressions of ACE2 receptors in gastrointestinal epithelial cells, diarrhoea had become the most common digestive symptom in COVID-19 patients [29, 30]. The replication of SARS-CoV-2 in the gastrointestinal tract should be given more attention in epidemic prevention to avoid its spread through the faecal-oral route.

Of all 375 imported cases from Russia through the Suifenhe port, the proportions of severe and critical patients were lower, accounting for 5.3% and 1.3%, respectively. Therefore, only approximately half of the patients received oxygen therapy, with nasal tube oxygen inhalation therapy accounting for the majority. The proportion of cases who received oxygen therapy in each group significantly increased with deterioration of the disease. Further analysis revealed that age, LYMPH, and LYM% were correlated to disease progression, with significantly elevated age and decreased levels of LYMPH and LYM% as the disease progressed. As a result, these factors can be used to determine disease severity in clinical practice.

The major limitation of the current study was the relatively small sample size, with inclusion of a total of 375 cases, all of which were imported from Russia, which may not represent the clinical features of all imported COVID-19 cases from overseas countries. Therefore, large-sample datasets of imported COVID-19 cases from different overseas countries are required to verify our findings. Our study is also limited by its retrospective nature.

### Countermeasures for imported COVID-19 cases from Russia through the Suifenhe port

The successful experiences in controlling domestic transmission of COVID-19 in China can be used for reference in imported cases from abroad. Controlling imported cases from overseas and preventing the second epidemic outbreak have posed new challenges in China [12]. Suifenhe city has established a joint prevention and control mechanism, namely “closed-loop management, segmented responsibility and seamless docking”, and has strictly carried out port quarantine measures of “three screenings, three inspections and one trans-shipment” to avoid the spread of overseas epidemics through the Suifenhe port, which is similar to the control measures adopted by some other countries [31, 32]. Among them, “three screenings” include three screening links of health declaration card, temperature monitoring, and medical patrolling; “three inspections” refer to the rigorous implementation of epidemiological, medical, and laboratory inspections; “one trans-shipment” means to transfer confirmed cases, suspected cases, close contacts and individuals with fever and respiratory symptoms to a designated hospital or a local joint prevention and control isolation program and generate handover records. “Six hundred percent” management and a control plan are strictly implemented, that is, 100% quarantine for entry vehicles, 100% temperature monitoring for entry personnel, 100% health declaration card verification, 100% nucleic acid amplification testing, 100% epidemiological investigation, and 100% centralized isolation. All entry personnel are sent to designated hotels for the isolation program to firmly cut off the source of infection. With the continuous upgrading of epidemic prevention and management measures, a large number of volunteers participate and play an important role.

RETRACTED

In accordance with the “four concentrations” principle, that is, concentration of patients, experts, medical resources and treatment, all confirmed cases were subjected to assessment, of whom asymptomatic infection cases, mild and moderate cases, and severe and critical cases were managed in the Suifenhe square cabin hospital, Mudanjiang Ankang hospital, and Hongqi Hospital Affiliated Mudanjiang Medical University, respectively. Eight transfer ambulances with negative pressure functions were deployed to complete the transfer of confirmed imported patients.

## Conclusions

To the best of our knowledge, our study presented the description of the latest and most comprehensive data on COVID-19 cases imported from Russia through the Suifenhe port and proposed corresponding countermeasures. Compared with domestic confirmed cases, these imported cases had significantly different clinical features. The results of the present study are practically and clinically significant for management and prevention of another outbreak of COVID-19. Certainly, the development of the epidemic is ever-changing, especially with the mutation of the virus. The prevention, diagnosis and treatment of COVID-19 also need to change to adapt to the development, but some basic principles should be consistent. The world is “a Community of a Shared Future for Mankind”. Therefore, it requires the joint efforts of all countries to overcome the pandemic.
